The article "NEK2 Serves as a Novel Biomarker and Enhances the Tumorigenicity of Clear-CellRenal-Cell Carcinoma by Activating WNT/β-Catenin Pathway" was retracted in 2023. Reasons: suspected computer-generated content; unreliable results or conclusions; lack of ethics approval or compliance; missing or withdrawn patient consent.

# NEK2 Serves as a Novel Biomarker and Enhances the Tumorigenicity of Clear-CellRenal-Cell Carcinoma by Activating WNT/*β*-Catenin Pathway

**DOI:** 10.1155/2022/1890823

**Published:** 2022-09-29

**Authors:** Jiancheng Zhou, Jiawei Lai, Yongyi Cheng, Weixing Qu

**Affiliations:** Department of Urology, Shaanxi Provincial People's Hospital, Xi'an 710068, Shaanxi, China

## Abstract

**Objective:**

Currently, cumulative evidence has shown that loss of NEK2 function suppresses tumor growth. However, complete studies on the regulatory role of NEK2 in clear-cellrenal-cell carcinoma (ccRCC) are rarely reported.

**Methods:**

The GEPIA database was used for information mining to analyze the gene expression differences between ccRCC tumor and normal tissues. At the same time, we analyzed the protein expression of NEK2 in clinical ccRCC samples and ccRCC cell lines. We detected the effect of NEK2 on the biological behavior of ccRCC at the cell level and further verified the biological effect of NEK2 on ccRCC cells in vivo by nude mouse tumorigenesis experiment. The expression of WNT/*β*-cateninpathway-related proteins and downstream proteins related to cell function were detected by Western blotting.

**Results:**

Using the GEPIA database, we observed that NEK2 expression level in ccRCC tissues was significantly higher than that in normal kidney tissues and was also related to tumor grade. The survival time of patients with ccRCC with high NEK2 expression was shorter than that of patients with low NEK2 expression. Compared with adjacent carcinoma and normal renal tubular epithelial cells, NEK2 levels were highly expressed in ccRCC tissues and ccRCC cell lines. NEK2 interference restrained ccRCC cell growth, migration, and invasion. NEK2 regulated the malignant behavior of ccRCC cells through the WNT/*β*-catenin pathway. Nude mouse tumorigenesis assay results showed that the transplanted tumors from NEK2 silenced mice grew more slowly and were smaller in size than those from control mice.

**Conclusions:**

NEK2 elevation may be associated with poor prognosis in ccRCC, and NEK2 enhances ccRCC cell proliferation, migration, and invasion ability by activating the WNT/*β*-catenin signaling pathway.

## 1. Introduction

Renal-cell carcinoma (RCC) is one of the ten most common malignant tumors in the world, and the incidence of RCC is second only to bladder cancer [1]. Clear-cellrenal-cell carcinoma (ccRCC) is the most common histological type of RCC, accounting for 75% of all renal cancers and the leading pathological type of death in renal cancer patients [2]. Therefore, it is of great significance to study the occurrence and development of ccRCC. Because clear-cellrenal-cell carcinoma is insensitive to both chemotherapy and radiotherapy, surgery is the preferred treatment for early renal cancer, and targeted therapy is the main treatment for advanced renal cancer [3]. Recently, with the development of targeted therapeutics, more and more targeted agents have been used in the clinical treatment of advanced or metastatic ccRCC. The results of clinical experiments showed that the targeted drugs significantly inhibited renal cancer cell growth and contributed to the improved prognosis of ccRCC patients [4]. But about 20% of patients treated with targeted drugs in the clinic will develop early resistance, resulting in poor treatment outcomes and poor patient outcomes [5–7]. There are studies statistically applying VEGF targeted agents to metastatic ccRCC with a median survival time of only 18.8 months [8, 9]. Therefore, it is important to elucidate the underlying molecular mechanisms of ccRCC progression and discover new highly effective and sensitive prognostic markers for the clinical diagnosis of ccRCC as well as develop new targeted therapeutics.

The article "NEK2 Serves as a Novel Biomarker and Enhances the Tumorigenicity of Clear-CellRenal-Cell Carcinoma by Activating WNT/β-Catenin Pathway" was retracted in 2023. Reasons: suspected computer-generated content; unreliable results or conclusions; lack of ethics approval or compliance; missing or withdrawn patient consent.

Never in mitosis gene A related kinase (NIMA) is a family of serine/threonine kinases representing NEK1-NEK11, located in the cytoplasm and mitochondria of ciliated centrosomes [10]. Accumulated evidence reveals that the NIMA-related kinase family (NEKs) is involved in various cellular functions and is associated with target pathways relevant to cancer development [11]. Thus, the members of NEKs have become drug targets of great interest. NEK2, a centrosomal serine/threonine kinase encoded by the NEK2 gene, is an essential enzyme in cell cycle progression, especially in mitotic regulation through the phosphorylation of different substrates [12]. NEK2 plays an important role in centrosome separation, microtubule organization, chromatin condensation, and the spindle assembly checkpoint. Upregulation of NEK2 leads to centrosome abnormalities and unipolar spindle formation and promotes aneuploidy by disrupting the control of mitotic checkpoints, leading to cell cycle disorders. [13, 14]. An increasing number of studies show that NEK2 expression is increased in tumor tissues, and NEK2 upregulation is closely associated with multiple types of tumor progression, drug resistance, and poor prognosis [15–17]. Meanwhile, a previous study demonstrated that deregulation of NEK2 protein is associated with poor prognosis in human ccRCC [18], but to date, there have been no reports on the regulatory mechanism of NEK2 protein on ccRCC.

In this study, we intend to detect the expression difference of NEK2 in ccRCC tissues and ccRCC cell lines, analyze the impact of NEK2 expression difference on the clinical prognosis of NEK2 patients, and finally explore the impact of NEK2 on the biological function of NEK2 in vivo and in vitro.

The article "NEK2 Serves as a Novel Biomarker and Enhances the Tumorigenicity of Clear-CellRenal-Cell Carcinoma by Activating WNT/β-Catenin Pathway" was retracted in 2023. Reasons: suspected computer-generated content; unreliable results or conclusions; lack of ethics approval or compliance; missing or withdrawn patient consent.

## 2. Materials and Methods

### 2.1. Patients and Tissue Specimens

In this study, 30 cases of clear-cellrenal-cell carcinoma (ccRCC) and adjacent noncancerous tissue specimens (normal tissues with the distance of 3 cm from the renal cancer tissues) removed by radical nephrectomy in Shaanxi Provincial People's Hospital from June 2016 and May 2020 were collected. All patients did not receive any radiotherapy, chemotherapy, or targeted therapy before the operation. Fresh ccRCC and adjacent noncancerous tissue specimens were collected during the operation, which was washed with PBS and immediately frozen in liquid nitrogen. Fresh ccRCC and adjacent noncancerous tissue specimens were collected intraoperatively and immediately frozen in liquid nitrogen after washing with PBS for Western blot analysis.

### 2.2. Cell Culture and Transfection

A498, Caki-1, and 786-O, as the most commonly used ccRCC cell lines and human proximal tubule epithelial cells (HK-2), were purchased from the cell resource center of the Shanghai Institutes of Biological Sciences, Chinese Academy of Sciences. 10% FBS was mixed with RPMI 1640 and then added into all cell plates and maintained in a 5% CO_2_ incubator at 37°C with 2–3 changes of medium per week. Subsequently, 786-O and Caki-1 cells in the logarithmic growth phase were harvested, digested and resuspended, and seeded in 6-well plates at 5 × 10^5^ cells/well and cultured overnight for cell transfection when the cell confluence reached approximately 80%. According to the Lipofectamine 2000 reagent instructions, shRNA targeting NEK2 (sh-NEK2: 5′-CCTGTATTGAGTGAGCTGAA-3′) and their negative control (sh-NC: 5′-TTCTCCGAACGTGTCACGT-3′) were transfected into the two cell lines, which were cultured for 48 h.

### 2.3. Western Blot Assay

ccRCC tissues and cells were collected and quickly loaded into 1.5 mL EP tubes with the addition of a well-configured RIPA lysis solution. The supernatant obtained by centrifugation after lysis was carefully aspirated, and the protein content was tested by the BAC method. Protein samples (20 *μ*g) were applied to 10% SDS-PAGE gels to separate and transferred to PVDF membranes by a wet rotation. The PVDF membranes were immersed in 5% nonfat milk powder sealant and sealed for 2 h. Reference to the recommended ratio in the instructions, 5% nonfat milk was used to dilute primary antibodies, including NEK2, E-cadherin, GAPDH, c-Myc, MMP-9, GSK3*β*, and *β*-catenin (1 : 1000) for overnight incubation at 4°C. After washing the membrane three times with TBST, the PVDF membranes were immersed in secondary antibody diluent and incubated for 1 h at room temperature on a shaker. Finally, the luminescent solution was prepared, and the protein bands were soaked slightly in the luminescent solution, put into the luminescent machine, and then, luminescence development was performed and pictures were retained by Image J software.

The article "NEK2 Serves as a Novel Biomarker and Enhances the Tumorigenicity of Clear-CellRenal-Cell Carcinoma by Activating WNT/β-Catenin Pathway" was retracted in 2023. Reasons: suspected computer-generated content; unreliable results or conclusions; lack of ethics approval or compliance; missing or withdrawn patient consent.

### 2.4. CCK-8 Assay

The cells were suspended in complete medium and the concentration of cell suspension was adjusted to 2 × 10^4^/mL. A uniform concentration of cell suspension (100 *μ*L/well) was seeded in 96-well plates. After seeding, the 96-well plates were incubated in a 5% CO_2_ incubator at a constant temperature for the corresponding planned time (24, 48, 72, and 96 h). At the planned assay time point, the 96-well plate was removed, 10 L of CCK-8 solution was added to the well of the cell to be tested, and continue to put the 96-well plate into the cell culture incubator for 1 h of incubation. Finally, the 96-well plate was removed, placed in the detection rack of the microplate reader, and the absorbance value (OD) of each well was detected at 450 nm.

### 2.5. 5-Ethynyl-2′-Deoxyuridine (EdU) Immunofluorescence Staining

EdU Kit (Ribobio) was utilized to assess cell proliferation. The 786-O and Caki-1 cells were suspended in complete medium and the concentration of cell suspension was adjusted to 1.5 × 10^5^/mL. A uniform concentration of cell suspension (200 *μ*L/well) was seeded into 48-well plates, and then 50 *μ*M of EdU marketing solution was added to each well to incubate with cells for 8 h. Subsequently, the cells were fixed with 70% ethanol, infiltrated with Triton X-100 and stained with Apollo reaction solution. After washing the cells three times with PBS, DAPI was used for nuclear staining. The images were captured under a fluorescence microscope (Olympus).

### 2.6. Cell Cycle Assay

Cell Cycle Staining Kit (MultiSciences Biotech Ltd., China) was utilized to cell cycle. 786-O and Caki-1 cells were suspended in complete medium and the concentration of cell suspension was adjusted to 5 × 10^5^ cells/mL. Ethanol at a concentration of 70% was added to the cultured cells for overnight fixation, subsequently, PBS was added to wash, and PI was added to avoid light staining for 30 min. Finally, the percentage of the cells in different phases was measured with flow cytometry.

### 2.7. Transwell Assays

After the serum-free medium and Matrigel were diluted at a ratio of 7 : 1 according to the instructions, they were evenly spread over the transwell upper chambers for invasion assays. For the migrated assay, the transwell upper chambers did not contain Matrigel. 786-O and Caki-1 cells (5 × 10^5^ cells/mL) were added to the upper chamber along with serum-free medium to 200 *μ*L. The lower chamber was then filled with 600 *μ*L of complete medium. After 24 h of incubation at 37°C in 5% CO_2_, the chambers were removed, and the cells on the Matrigel were gently wiped off using a cotton swab, and the PBS working solution was used to wash chambers repeatedly three times. The chambers were then fixed in 4% paraformaldehyde for 20 min, and washed repeatedly three times with PBS working solution. Next, after staining with crystal violet dye solution for 20 min, the chambers were washed repeatedly thrice with PBS and left to air dry at room temperature. Eventually, the number of invaded or migrated cells within five random fields was counted under an IX51 microscope.

The article "NEK2 Serves as a Novel Biomarker and Enhances the Tumorigenicity of Clear-CellRenal-Cell Carcinoma by Activating WNT/β-Catenin Pathway" was retracted in 2023. Reasons: suspected computer-generated content; unreliable results or conclusions; lack of ethics approval or compliance; missing or withdrawn patient consent.

### 2.8. Immunohistochemistry

Tissue samples of 5 *μ*m-thick paraffin sections were conventionally dewaxed, dehydrated by gradient ethanol, repaired with EDTA (pH = 9.0) for 3 min, sealed with 3% methanol hydrogen peroxide, and added with Ki67 primary antibody (1 : 200) at 4°C overnight. Next, slides were incubated with HRP-secondary antibodies, visualized with DAB, counterstained with hematoxylin, routinely dehydrated, and transparent. Images were captured by a light microscope.

### 2.9. Animal Experiments

Twenty BALB/c nude mice (5-week-old, 15–22 g) were purchased from the experimental Animal Center of Xi'an Jiaotong University, which were randomly divided into sh-NEK2 and sh-NC groups. 786-O cells transfected with sh-NEK2 or sh-NC were resuspended with PBS, and the cell concentration was adjusted to 3 × 10^7^ cells/mL. 100 L of the above cell suspension was respectively pipetted and subcutaneously injected into the left axilla of mice. Nude mice status and subcutaneous tumorigenesis were observed weekly after inoculation. Six weeks after tumor formation, the nude mice were sacrificed to exfoliate the tumor, and the tumor was tested and weighed. Tumor volumes were calculated according to the formula: [length × width^2^]/2. Part of the tumor was stored in formalin for immunohistochemical experiments.

### 2.10. Statistical Analysis

The results of the measurement data were expressed as mean ± standard deviation (SD) from three independent experiments. The Shapiro –Wilk test was utilized to verify that the measurement data were normally distributed. The *t*-test was applied to compare the measurement data in accordance with normal distribution. SPSS 20.0 was used for data analysis. *P* < 0.05 considered that the difference was statistically significant.

## 3. Results

### 3.1. The Expression of NEK2 Was Overexpressed in ccRCC and Correlated with Clinical Parameters

NEK2 has been reported to play an oncogene role in other tumors. Thus, we want to further study its role in ccRCC progression. Using the GEPIA database, we found that NEK2 expression was upregulated in kidney clear renal cell carcinoma (KIRC) tumor tissues (Figure 1(a)). Surprisingly, compared with stages III and IV, the expression of NEK2 was remarkably differentially expressed in TNM stages I and II (Figure 1(b)). The results of the GEPIA database also revealed that elevated NEK2 was negatively correlated with the shortening of overall survival and disease-free survival (Figures 1(c) and 1(d)). To study whether the levels of NEK2 in ccRCC patients were consistent with the results of bioinformatics analysis, we collected 30 pairs of ccRCC tissues and adjacent noncancerous tissues to estimate NEK2 expression by Western blotting. The results revealed that a high level of NEK2 was found in ccRCC tissues (Figure 1(e)). Subsequently, we also demonstrated that NEK2 was elevated in ccRCC cell lines (A498, Caki-1, and 786-O) in comparison with the human proximal tubule epithelial cell line HK-2 (Figure 1(f)).

The article "NEK2 Serves as a Novel Biomarker and Enhances the Tumorigenicity of Clear-CellRenal-Cell Carcinoma by Activating WNT/β-Catenin Pathway" was retracted in 2023. Reasons: suspected computer-generated content; unreliable results or conclusions; lack of ethics approval or compliance; missing or withdrawn patient consent.

### 3.2. Interference of NEK2 Reduced ccRCC Cell Growth and Induced Cell Cycle Arrest

To investigate whether NEK2 regulated the malignant biological behavior of ccRCC cells, we constructed sh-NEK2 or sh-NC and transfected them into 786-O and Caki-1 cells and then used them for subsequent experiments. Western blotting confirmed that NEK2 protein expression was effectively decreased in sh-NEK2 transfected cells (Figure 2(a)). CCK-8 assays indicated that the inhibition of NEK2 by sh-NEK2 prominently impaired 786-O and Caki-1 cell proliferation (Figure 2(b)). Similarly, the sh-NEK2 group had fewer cell proliferation than the sh-NC group, as demonstrated by the EDU assay (Figure 2(c)). Through flow cytometry, we demonstrated that NEK2 silencing resulted in prominently increased cell cycle arrest at the G0/G1 stage and prominently decreased cell cycle arrest at the S phase (Figure 2(d)).

### 3.3. Knockdown of NEK2 Reduced Migration and Invasion of ccRCC Cells

Through the analysis of the GEPIA database, we found that the elevation of NEK2 was prominently correlated with the prognosis and TNM stage of ccRCC. Therefore, we speculated that NEK2 may have a hand in the invasion and metastasis of ccRCC. We first examined the effect of NEK2 on the migration of ccRCC cells in vitro. In 786-O and Caki-1 cells, the migration ability of cells was significantly decreased, and NEK2 silencing triggered a decline in the number of cells passing through the chamber (Figure 3(a)). Transwell assays further demonstrated that NEK2 interference effectively suppressed the invasion ability of cells and caused a marked decrease in the number of invaded cells (Figure 3(b)). Of note, MMP-9 and E-cadherin are key factors in tumor invasion and metastasis. To investigate whether MMP-9 and E-cadherin participate in the invasion and migration of ccRCC promoted by NEK2, we detected MMP-9 and E-cadherin levels in NEK2 silenced cells and negative control cells. As predicted, the results of Western blotting indicated that NEK2 silencing prominently augmented the E-cadherin protein level and remarkably reduced the MMP-9 protein level (Figures 3(c) and 3(d)).

The article "NEK2 Serves as a Novel Biomarker and Enhances the Tumorigenicity of Clear-CellRenal-Cell Carcinoma by Activating WNT/β-Catenin Pathway" was retracted in 2023. Reasons: suspected computer-generated content; unreliable results or conclusions; lack of ethics approval or compliance; missing or withdrawn patient consent.

### 3.4. NEK2 Was Involved in the Malignant Behavior of ccRCC Cells via Wnt/*β*-Catenin Pathway

After confirming that NEK2 can affect the biological behavior of ccRCC, we further investigated the signaling pathway in which NEK2 may be involved. The Wnt/*β*-catenin signaling pathway has been reported to regulate ccRCC progression [19–21]. To determine whether NEK2 modulated the Wnt/*β*-catenin pathway to enhance the malignant behavior of clear-cellrenal-cell carcinoma, WNT pathway-related protein levels, including GSK3*β*, *β*-catenin, and c-Myc, in NEK2-depleted 786-O and Caki-1 cells and negative control cells were tested by Western blotting. The results demonstrated that the expression of phosphorylated GSK3*β*, *β*-catenin, and c-Myc was decreased (Figures 4(a)–4(c)).

### 3.5. Knockdown of NEK2 Restrained Tumor Growth In Vivo

To further validate the effect of NEK2 on ccRCC, we performed subcutaneous tumorigenesis in nude mice by applying the constructed 786-O cells with stable interference of NEK2 and the negative control cells to observe the tumor cell growth in vivo. The results uncovered that NEK2 interference resulted in inhibition of tumor growth, as demonstrated by a significant reduction in tumor size and weight in mice (Figures 5(a)–5(c)). Western blotting indicated that the NEK2 level in tumor tissues was abated in the sh-NEK2 group (Figure 5(d)). Of note, immunohistochemical analysis of Ki67 levels in tissues from tumors displayed that the sh-NEK2 group exhibited an effectively reduced Ki67 expression intensity in comparison with the sh-NC group (Figure 5(e)).

## 4. Discussion

In the current work, using bioinformatics analysis, we found that NEK2 expression was higher in ccRCC tissues than in adjacent noncancerous tissues. Furthermore, the results of survival analysis showed that patients with ccRCC in the NEK2 high-expression group had a significantly shorter survival time than patients with ccRCC in the NEK2 low-expression group. At the same time, the level of NEK2 protein expression in ccRCC tissues using Western blot analysis suggested that NEK2 protein expression was elevated in ccRCC tissues, and these results were consistent with the previous information analysis. We simultaneously examined NEK2 protein levels in ccRCC cell lines, namely, 786-O, Caki-1, A-498, and HK-2 cells, and the results suggested that NEK2 was more highly expressed in ccRCC cell lines than in HK-2 cells and that NEK2 expression was effectively increased in ccRCC cell lines, which also further corroborated previous examinations at the cellular and tissue levels.

The article "NEK2 Serves as a Novel Biomarker and Enhances the Tumorigenicity of Clear-CellRenal-Cell Carcinoma by Activating WNT/β-Catenin Pathway" was retracted in 2023. Reasons: suspected computer-generated content; unreliable results or conclusions; lack of ethics approval or compliance; missing or withdrawn patient consent.

Previous studies have identified abnormal levels of NEK2 proteins in a series of tumors, and NEK2 is involved in cell growth and apoptosis, enhances the ability of tumor invasion, and reduces the sensitivity of tumor cells to chemotherapeutic agents, thereby contributing to the tumorigenic capacity of malignant tumors [22, 23]. Through the inactivation of the AKT pathway, NEK2 silencing hindered gastric cancer cell growth by inducing autophagic cell death and suppressing aerobic glycolysis [24]. In the study of NSCLC, NEK2 not only mediated tumor angiogenesis and M2 polarization of macrophages but also contributes to tumor cell proliferation and invasion, thus promoting the occurrence of nonsmall-cell lung cancer [25]. TP53 deletion elevated NEK2 expression by inducing NEK2 amplification, thereby inhibiting the ability of proliferation, drug resistance development, and tumorigenesis of multiple myeloma cells [26]. Given the above, NEK2 may serve as a molecular target in ccRCC research. In this study, we constructed NEK2 knockdown cells and xenotransplantation tumor models and conducted cell function and animal experiments after confirming their stable expression. Knockdown of NEK2 resulted in retarded ccRCC cell growth and significantly decreased cell migration and invasion abilities. Besides, NEK2 knockdown clearly inhibited tumor cell growth in vivo with reduced tumorigenic capacity.

WNT/*β*-catenin is a class of signaling pathways that have been highly conserved across species evolution and that play an important role in embryogenesis, organ formation, and regulation of homeostasis [27, 28]. Much tumorigenesis and progression are associated with mutations in key proteins in this signaling pathway, leading to aberrant activation of signaling. WNT proteins, through their interaction with cell surface specific receptors, cause the accumulation of *β*-catenin proteins in the cytoplasm, ultimately leading to the proliferation and metastasis of cancer cells [29]. *β*-Catenin protein has various cellular functions, where it can interact with E-cadherin at cell junctions, thereby playing an adhesive role [30]. Additionally, MMP-9 is one of the Wnt pathway target genes, which can be transcriptionally regulated [31]. According to some substantial studies, the WNT/*β*-catenin pathway is hyperactivated in ccRCC, and targeted inhibition of the WNT/*β*-catenin pathway may become a feasible therapeutic strategy for tumors [32–34]. Here, our results showed that NEK2 silencing could obviously downregulate the protein expression levels of key proteins, such as p-GSK-3*β*, *β*-catenin, and the downstream regulator c-Myc, proving that NEK2 silencing could inhibit the WNT/*β*-catenin signaling pathway.

The article "NEK2 Serves as a Novel Biomarker and Enhances the Tumorigenicity of Clear-CellRenal-Cell Carcinoma by Activating WNT/β-Catenin Pathway" was retracted in 2023. Reasons: suspected computer-generated content; unreliable results or conclusions; lack of ethics approval or compliance; missing or withdrawn patient consent.

In conclusion, NEK2 was upregulated in ccRCC tumors, and the degree of expression is closely related to tumor prognosis, which may provide a basis for early diagnosis and prognosis. NEK2 interference obviously repressed ccRCC cell growth and concurrently restrained invasion and migration. On a mechanistic level, our results suggest that NEK2 may act by repressing Wnt/*β*-catenin pathway to suppress ccRCC growth. The result of this experiment will provide insight into the molecular mechanism of NEK2 in ccRCC and lay a foundation for further exploration of it as a candidate for the therapy of ccRCC.

## Figures and Tables

**Figure 1:** Elevated NEK2 was found in ccRCC tissues and cell lines. (a): NEK2 expression was predicted in kidney clear renal cell carcinoma (KIRC) samples and normal sample by the GEPIA database. (b): NEK2 expressions at TNM stages I, II, III, and IV were predicted by the GEPIA database. (c, d) Overall survival and progression-free survival of ccRCC patients with high or low expression of NEK2 was predicted by the GEPIA database. (e) NEK2 expression in tumor and adjacent issues collected from ccRCC patients (*n* = 30). (f): NEK2 expression in 786-O, Caki-1 and A498, and HK-2 cells. ^*∗*^*P* < 0.05.

**Figure 2:** NEK2 silencing restrained cell growth. (a) Western blotting detection of NEK2 level in ccRCC cells after transfection. (b, c) CCK-8 and EDU assays detection of ccRCC cell proliferation after transfection. (d) Flow cytometry detection of the ccRCC cell cycle after transfection. ^*∗*^*P* < 0.05.

**Figure 3:** NEK2 silencing restrained ccRCC cell migration and invasion. sh-NEK2 or sh-NC was transfected into 786-O and Caki-1 cells, respectively. (a) Transwell migration assay detection of ccRCC cell migration. Scale bar: 100 *μ*m. (b) Transwell invasion assay detection of ccRCC cell invasion. Scale bar: 100 *μ*m. (c) Western blotting detection of E-cadherin in ccRCC cells. (d) Western blotting detection of E-cadherin and MMP-9 level in ccRCC cells. ^*∗*^*P* < 0.05.

**Figure 4:** NEK2 silencing blocked Wnt/*β*-catenin pathway activation. sh-NEK2 or sh-NC was transfected into 786-O and Caki-1 cells, respectively. (a–c) Western blotting detection of WNT pathway-related protein (GSK3*β*, *β*-catenin, and c-Myc) level in ccRCC cells after transfection. ^*∗*^*P* < 0.05.

The article "NEK2 Serves as a Novel Biomarker and Enhances the Tumorigenicity of Clear-CellRenal-Cell Carcinoma by Activating WNT/β-Catenin Pathway" was retracted in 2023. Reasons: suspected computer-generated content; unreliable results or conclusions; lack of ethics approval or compliance; missing or withdrawn patient consent.

**Figure 5:** NEK2 silencing restrained cell growth in ccRCC in vivo. NEK2 stable knockdown (sh-NEK2) and negative control (sh-NC) 786-O cells were utilized to construct a xenograft model in mice. (a) Observation of tumor growth following NEK2 interference. (b) Detection of mouse tumor volume following NEK2 interference. (c) Detection of mouse tumor weight following NEK2 interference. (d, e) Western blotting detection of NEK2 level following NEK2 interference. (e) Immunohistochemical detection of Ki67 level following NEK2 interference. ^*∗*^*P* < 0.05.

## Data Availability

The labeled dataset used to support the findings of this study are available from the corresponding author upon request.
